The article "Bone mesenchymal stem cell-derived exosomal microRNA-29b-3p prevents hypoxic-ischemic injury in rat brain by activating the PTEN-mediated Akt signaling pathway" was retracted in 2020. Reasons: results that could not be reproduced; unreliable results or conclusions.

# Bone mesenchymal stem cell-derived exosomal microRNA-29b-3p prevents hypoxic-ischemic injury in rat brain by activating the PTEN-mediated Akt signaling pathway

**DOI:** 10.1186/s12974-020-1725-8

**Published:** 2020-02-03

**Authors:** Kun Hou, Guichen Li, Jinchuan Zhao, Baofeng Xu, Yang Zhang, Jinlu Yu, Kan Xu

**Affiliations:** 1 Department of Neurosurgery, The First Hospital of Jilin University, No. 1 Xinmin Avenue, Changchun, 130021 Jilin People’s Republic of China; 2 Department of Neurology, The First Hospital of Jilin University, Changchun, 130021 People’s Republic of China

**Keywords:** Hypoxic-ischemic brain injury, microRNA-29b-3p, Bone mesenchymal stem cells, Angiogenesis, Exosome, PTEN, Akt signaling pathway

## Abstract

**Background:**

Mesenchymal stem cells (MSCs) are suspected to exert neuroprotective effects in brain injury, in part through the secretion of extracellular vesicles like exosomes containing bioactive compounds. We now investigate the mechanism by which bone marrow MSCs (BMSCs)-derived exosomes harboring the small non-coding RNA miR-29b-3p protect against hypoxic-ischemic brain injury in rats.

**Methods:**

We established a rat model of middle cerebral artery occlusion (MCAO) and primary cortical neuron or brain microvascular endothelial cell (BMEC) models of oxygen and glucose deprivation (OGD). Exosomes were isolated from the culture medium of BMSCs. We treated the MCAO rats with BMSC-derived exosomes in vivo, and likewise the OGD-treated neurons and BMECs in vitro. We then measured apoptosis- and angiogenesis-related features using TUNEL and CD31 immunohistochemical staining and in vitro Matrigel angiogenesis assays.

**Results:**

The dual luciferase reporter gene assay showed that miR-29b-3p targeted the protein phosphatase and tensin homolog (PTEN). miR-29b-3p was downregulated and PTEN was upregulated in the brain of MCAO rats and in OGD-treated cultured neurons. MCAO rats and OGD-treated neurons showed promoted apoptosis and decreased angiogenesis, but overexpression of miR-29b-3p or silencing of PTEN could reverse these alterations. Furthermore, miR-29b-3p could negatively regulate PTEN and activate the Akt signaling pathway. BMSCs-derived exosomes also exerted protective effects against apoptosis of OGD neurons and cell apoptosis in the brain samples from MCAO rats, where we also observed promotion of angiogenesis.

**Conclusion:**

BMSC-derived exosomal miR-29b-3p ameliorates ischemic brain injury by promoting angiogenesis and suppressing neuronal apoptosis, a finding which may be of great significance in the treatment of hypoxic-ischemic brain injury.

## Background

Stroke is a common neurological disease that often leads to persistent disability, and is the third most common cause of death worldwide [1]. Acute ischemic stroke, which accounts for more than 80% of all stroke cases, may result in permanent brain damage when restoration of circulation is delayed [2]. Most cases of cerebral stroke result from transient or permanent occlusion of a cerebral blood vessel, which eventually proceeds to brain infarction [3]. Nowadays, the first-line treatment for ischemic stroke is thrombolysis with intravenous tissue plasminogen activator. However, the restoration of blood flow may under certain circumstances exacerbate oxidative stress and inflammatory responses [4, 5]. Therefore, there is an urgent need for innovative stroke treatments.

The article "Bone mesenchymal stem cell-derived exosomal microRNA-29b-3p prevents hypoxic-ischemic injury in rat brain by activating the PTEN-mediated Akt signaling pathway" was retracted in 2020. Reasons: results that could not be reproduced; unreliable results or conclusions.

It is well-recognized that the route to hypoxic-ischemic brain injury is a complicated process involving various biological pathways both in the early and late stages [6]. Among the involved pathways, angiogenesis and neurogenesis are now principal targets in the treatment of stroke [7]. Transplantation with mesenchymal stem cells (MSCs) is reportedly a candidate target in the treatment of neonatal hypoxic-ischemic brain injury, and is increasingly drawing the attention of stroke researchers [8]. The exosomes derived from MSCs mediate the therapeutic actions of MSCs [9, 10]. In recent years, growing evidence has suggested that microRNAs (miRNAs) play critical roles in ischemic stroke [11]. Experimental therapeutic approaches based on miRNAs have been developed to help post-stroke neurological recovery and ameliorate ischemic brain injury [12, 13]. miR-29b-3p, one of the members of the miR-29b family to be identified, exhibits therapeutic potential for treating cardiometabolic disorders [14]. Furthermore, the expression of miR-29b-3p was reduced in patients with intestinal ischemia-reperfusion injury [15]. The gene for phosphatase and tensin homolog (PETN), which is located on human chromosome 19, encodes a dual phosphatase enzyme that dephosphorylates both protein and lipid substrates [16]. Also, PTEN is a negative regulator of the phosphatidylinositol 3-kinase/protein kinase B (PI3K/Akt) signaling pathway [17], which is implicated in hypoxic-ischemic injury [18]. However, it has been unclear whether bone marrow mesenchymal stem cells (BMSCs)-derived exosomes and miR-29b-3p moderate the severity of ischemic brain injury and whether their regulation is dependent on PTEN or the Akt signaling pathway. Given that PTEN regulates angiogenesis in tumors and healthy tissues, it is notable that angiogenesis of brain microvascular endothelial cells (BMECs) is necessary for the functional restoration of brain injury, such as ischemic stroke [19]. Therefore, we conducted extensive experiments to test the hypothesis that BMSC-derived exosomal miR-29b-3p participates in the neuronal apoptosis and angiogenesis of BMECs in the context of hypoxic-ischemic brain injury, which might be associated with PTEN and the Akt signaling pathway.

The article "Bone mesenchymal stem cell-derived exosomal microRNA-29b-3p prevents hypoxic-ischemic injury in rat brain by activating the PTEN-mediated Akt signaling pathway" was retracted in 2020. Reasons: results that could not be reproduced; unreliable results or conclusions.

## Materials and methods

### Ethics statement

The present study was approved by the Ethics Committee of The First Hospital of Jilin University. All procedures involving animals were conducted in line with the regulations of the institutional animal care and use committee (ethics number: 2018-415).

### Rat middle cerebral artery occlusion model establishment and neurobehavioral evaluation

A permanent model of middle cerebral artery occlusion (MCAO) was established according to the previously reported Longa method [20, 21], using 32 male Sprague-Dawley (SD) rats (aged 6–8 weeks, initial weight 200 ± 15 g, Shanghai Sippr Bk Laboratory Animals Co., Ltd., Shanghai, China) as previously reported [22]. The rats used in the experiment were housed under specific-pathogen-free (SPF) conditions in a 12-h light/dark cycle, with free access to food and water. The MCAO procedure was applied only when the rats reached a body weight of 250 ± 12 g. Then, a thread plug was prepared with a 27-mm-long 3–0 nylon thread. The tip was heated on an alcohol burner to form a plug of hemispherical bulb shape with a diameter of 0.33 mm, which was smeared with silicone grease. Rats were anesthetized with 2% pentobarbital sodium at a dose of 30 mg/kg (i.p.) before they were fixed on the operating table in the supine position. The right common carotid artery (CCA), internal carotid artery (ICA), and external carotid artery (ECA) were separated. The ECA and CCA were ligated. After clamping the distal end of the ICA, a cut was quickly made at the bifurcation of ECA and ICA. The nylon thread (a mark was made 2 cm from the heated bulb end) was inserted from the incision into the ICA. The nylon thread and the ICA were ligated slightly at the incision. Then, the arterial clamp that clamped the ICA was loosened. The nylon thread was continued to be inserted until a slight resistance was felt (the insertion depth was about 18.5 ± 0.5 mm), and it was pulled out slightly. Thus, cerebral ischemia was developed due to middle cerebral artery occlusion. The neurological state of the MCAO rats was assessed within 1–2 h upon they awakened from anesthesia (about 30 min after operation). According to Bederson’s behavioral scoring method [23], the neurological function of the rats was evaluated by a double-blind scoring method, as follows: (1) no central nervous system injury symptoms (0 point); (2) unable to fully extend the contralateral front claw (1 point); (3) circling toward the side opposite the surgery (2 points); (4) falling to the side away from the surgery (3 points); (5) unable to walk spontaneously or failure to regain consciousness (4 points). A total of 32 rats were used for modeling, and the rats with scores in the range of 1–3 were regarded as successfully modeled MCAO rats (28/32; 87.5%), and the others were excluded from the subsequent experiments. The successfully modeled rats were randomly assigned into four groups (*n* = 7 in each group). Rats assigned to the sham group (*n* = 7) were subjected to the procedures of isolating carotid arteries, but without the insertion of a nylon thread.

The article "Bone mesenchymal stem cell-derived exosomal microRNA-29b-3p prevents hypoxic-ischemic injury in rat brain by activating the PTEN-mediated Akt signaling pathway" was retracted in 2020. Reasons: results that could not be reproduced; unreliable results or conclusions.

Intracerebroventricular stereotactic injection of MSCs-derived exosome (MSCs-Exo) or MSCs-Exo-miR-29b-3p agomir at lateral ventricle was carried out 2 h after the MCAO model was first developed, i.e., immediately after behavioral assessment. Rats were anesthetized as above mentioned, whereupon their heads were fixed on the stereotaxic instrument. Then, hair on the scalp was removed, and the skin was disinfected with iodophor and 75% alcohol. An incision measuring 1.5 cm was cut along the midline of the head to expose the skull around the Bregma. According to the stereotactic atlas of the rat, a trocar was inserted into the lateral ventricle (0.8 mm posterior to the Bregma, 1.5 mm next to the midline, 4.0 mm below the outer surface of the skull) [21]. The trocar was reserved for further use. The rats were placed in a warmed box with free access to food and water. One week later, the rats were administered by trocar. An indwelling needle was reserved for future use. The MSCs-Exo or MSCs-Exo-miR-29b-3p agomir was injected one time every day for 3 days at a dose of 100 μg/kg/day [24]. After another 72 h, the rats were euthanized, and the brains were collected and divided into portions used for 2,3,5-triphenyl tetrazolium chloride (TTC) staining, immunohistochemistry, as well as RNA and protein isolation.

### Isolation of primary cortical neurons, BMECs and BMSCs

Primary cortical neurons were isolated from the cerebral cortices under SPF conditions of fetal rats aged 16–18 days using a modification of Yavin’s method [25]. Then the isolated cortices were cut into small pieces, mixed with Dulbecco’s modified Eagle’s medium (DMEM), and transferred to a sterile culture bottle, followed by trituration with a pasteurized tube 30 times. Next, the suspension was subjected to centrifugation at 1000 g for 5 min. The isolated cells were cultured at 37 °C with 5% CO_2_ at a density of 1 × 10^6^ cells/well on culture plates which had been coated with 50 μg/mL poly-*L*-lysine prior to use. After incubation for 4 h, the medium was renewed with neuron-specific culture medium. Finally, the growth of the cells was observed under a microscope.

The article "Bone mesenchymal stem cell-derived exosomal microRNA-29b-3p prevents hypoxic-ischemic injury in rat brain by activating the PTEN-mediated Akt signaling pathway" was retracted in 2020. Reasons: results that could not be reproduced; unreliable results or conclusions.

For BMEC isolation, the SD rats (aged 6–8 weeks, weighing 200–250 g) were euthanized by intraperitoneal injection of an overdose of pentobarbital sodium (6%, 90 mg/kg). The cerebral cortex was dissected and immersed in cold D-Hanks and DMEM. The tissues were cut into pieces and water-bathed with 0.1% type II collagenase for 1.5 h. After centrifugation at 1000 g at room temperature for 8 min, the tissue blocks were suspended in 20% bovine serum albumin (BSA) and centrifuged at 1000 g at 4 °C for 20 min. Then the tissue blocks were water-bathed again with 0.1% collagenase/dispase at 37 °C for 1 h. After a recentrifugation at 1000 g at room temperature for 8 min, the tissue blocks were resuspended in 2 mL DMEM and coated with 12 mL 50% Percoll. The microvascular segments were removed by centrifugation twice with DMEM at 1000 g at room temperature for 5 min. The obtained pellets were suspended in DMEM complete culture medium, seeded in culture dishes pre-coated with gelatin substrate, and cultured in an incubator with 5% CO_2_ at 37 °C. After 24 h, the medium was changed with fresh medium supplemented with 1 ng/mL brain fibroblast growth factor. Every other day, the medium was renewed. Cells at passage three were used for animal experiments and exosome isolation.

Adult male SD rats (aged 6–8 weeks, weighing 200–250 g) were euthanized as above and bone marrow was obtained by rinsing the fractured femur of rats with DMEM (Hyclone, Marlborough, MA, USA) containing 10% fetal bovine serum (FBS). The marrow cells were cultured in DMEM containing 10% FBS plus 1% penicillin-streptomycin (P1400, Solarbio, Beijing, China) and detached with 0.25% trypsin plus ethylene diamine tetraacetic acid (concentration). The culture media were ultra-centrifugated at 120,000 g at 4 °C for 2 h to isolate the serum exosomes before use.

### Neuron oxygen-glucose deprivation model

We performed the oxygen-glucose deprivation (OGD) treatment in rat primary cortical neurons and BMECs as previously reported [22]. For OGD treatment, the culture medium was renewed with ischemic-mimetic D-Hanks containing 140 mM NaCl, 3.5 mM KCl, 0.43 mM KH_2_PO_4_, 1.25 mM MgSO_4_, 1.7 mM CaCl_2_, 5 mM NaHCO_3_, and 20 mM N-2-hydroxyethylpiperazine-N′-2-ethanesulfonic acid (pH = 7.2–7.4). Then cells were cultured in a hypoxic incubator supplemented with 95% N_2_/5% CO_2_ for 6 h at 37 °C (Billups-Rothenberg, San Diego, CA, USA) and collected immediately thereafter [26, 27].

### Cell transfection

When the BMSCs had reached 80–90% confluence, the cells were transfected according to the instructions for Lipofectamine 2000 (11668-019, Invitrogen, New York, CA, USA). Group 1: negative control (NC) mimic group (BMSCs treated with NC mimic), miR-29b-3p mimic group (BMSCs treated with miR-29b-3p mimic), NC inhibitor group (BMSCs treated with NC inhibitor), and miR-29b-3p inhibitor group (BMSCs treated with miR-29b-3p inhibitor). Group 2: OGD + BMSCs + miR-29b-3p mimic NC group (OGD cells co-cultured with exosome of BMSCs treated with NC mimic), OGD + BMSCs + miR-29b-3p mimic group (OGD cells co-cultured with exosome of BMSCs treated with miR-29b-3p mimic), OGD + BMSCs + miR-29b-3p inhibitor NC group (OGD cells co-cultured with exosome of BMSCs treated with miR-29b-3p inhibitor NC), and OGD + BMSCs + miR-29b-3p inhibitor group (OGD cells transfected with exosome of BMSCs treated with miR-29b-3p inhibitor). The mimic and inhibitor of miR-29b-3p were purchased from Ribobio Company (https://www.ribobio.com/) and transfected at a concentration of 100 nM.

The article "Bone mesenchymal stem cell-derived exosomal microRNA-29b-3p prevents hypoxic-ischemic injury in rat brain by activating the PTEN-mediated Akt signaling pathway" was retracted in 2020. Reasons: results that could not be reproduced; unreliable results or conclusions.

### Lentivirus construction and infection

The lentiviruses harboring miR-29b-3p overexpression and shRNA targeting PTEN were purchased from Genechem (Shanghai, China). Neurons or endothelial cells were infected with lentivirus. The subsequent experiments were carried out 24 h after infection.

### Extraction, identification, and labeling of exosomes

BMSCs-derived exosomes were extracted as previously reported [28], and the morphology and size distribution of exosomes were observed by transmission electron microscopy and dynamic light scattering (DLS) analysis. The exosome markers were assessed by Western blot analysis. PKH-67 labelling was performed following the PKH-67 kit instructions (MINI61-KT, Sigma-Aldrich, St. Louis, MO, USA). In brief, the exosome was incubated with PKH67-Diluent C for 5 min, and the staining was terminated with 0.5% BSA. Then the exosome was purified with the exosome extraction kit and the PKH-67-labeled exosome was obtained. Neurons and BMECs were incubated with PKH-67-labeled exosomes for 24 h. After being fixed in 4% paraformaldehyde at room temperature for 30 min, cells were stained by 4′,6-diamidino-2-phenylindole 2hci (DAPI; 36308ES11, Yeasen Biotechnology Co., Ltd., Shanghai, China) for 5 min, followed by observation under an inverted fluorescence microscopy (DMi8, Leica, Wetzlar, Germany) and photographed.

### TTC staining

The brain tissues were obtained from rats (*n* = 7 in each group) and cut onto 1-mm-thick sections. TTC solution (2%, T8170, Solarbio, Beijing, China) was added to the brain tissue sections for a 10–15-min incubation at 37 °C, and the sections were fixed using 4% paraformaldehyde, observed microscopically, and analyzed with the ImageJ software.

The article "Bone mesenchymal stem cell-derived exosomal microRNA-29b-3p prevents hypoxic-ischemic injury in rat brain by activating the PTEN-mediated Akt signaling pathway" was retracted in 2020. Reasons: results that could not be reproduced; unreliable results or conclusions.

### Terminal deoxyribonucleotidyl transferase-mediated biotin-16-dUTP nick-end labelling assay

The apoptosis of tissues was evaluated following the cell apoptosis detection kit instructions (TUN11684817, Roche, Mannheim, Germany). The tissue sections were dewaxed, rehydrated, and pretreated with protease-K for 30 min, followed by terminal deoxynucleotidyl transferase dUTP nick end labeling (TUNEL) staining for apoptosis detection at 37 °C for 1 h. Converter-pod was added to the sections followed by incubation at 37 °C for 30 min, and washing with phosphate-buffered saline (PBS), incubation with diaminobenzidine for 10 min. The sections were then counter-stained with hematoxylin, rinsed, dehydrated, and sealed. With a drop of PBS or glycerin placed in the field of vision, apoptotic cells (200–500 cells) were observed and photographed by optical microscopy (IX53, Olympus Optical Co., Ltd., Tokyo, Japan). We judged the morphological characteristics of the apoptotic cells; un-stained cells were small with intact membrane but with the foaming phenomenon, whose apoptotic bodies first appear at a late stage, with the adherent cells being crumpled, rounded, and felling off. The stained cells exhibit chromatin condensation, with marginalization and lysed nuclear membranes, and with chromatin divided into masses/apoptotic bodies. Five sections of each rat brain sample were randomly selected for assessment.

The pre-treatment of the cultured cells was conducted as follows: the slides were coated with a thin layer of polylysine, air-dried, rinsed in deionized water, and stored at 4 °C. Apoptosis was induced by the appropriate method, and there was a negative control (NC) group without induction of cell apoptosis. About 1 × 10^6^ cells were collected by centrifugation, washed in PBS, resuspended, transferred to the coated slides, and air-dried. The slides were then fixed in 4% paraformaldehyde for 25 min and treated with 0.2% Triton X-100 for 5 min, with subsequent procedures the same as those for paraffin-embedded section.

### RNA isolation and reverse transcription quantitative polymerase chain reaction

Total RNA from cells and tissues, and exosome-derived RNA were extracted using TRIZOL (15596-018, Beijing Solabio Life Sciences Co., Ltd., Beijing, China). The primers used in this study were synthesized by Takara Company (Dalian, Liaoning, China) (Table 1). Using GAPDH and U6 as internal reference primers, the relative mRNA expression of target genes was calculated by the 2^-△△Ct^ method [29].

**Table 1:** Primer sequence for RT-qPCR

miRNA/mRNA	Sequence (5′-3′)	
miR-29b-3p	F: TTCCTATGCATATACTTCT	R: CGTATCCAGTGCGAATA
PTEN	F: ATCTTGTGCTCACCCTGACA	R: ACCTCTCGGGAGTACACACT
GAPDH	F: CTGACATGCCGCCTGGAGA	R: ATGTAGGCCATGAGGTCCAC
U6	F: ATGACGTCTGCCTTGGAGAAC	R: TCAGTGTGCTACGGAGTTCAG
Bcl-2	F: AGCCCTGTGCCACCTGTGGT	R: ACTGGACATCTCTGCAAAGTCGCG
Bax	F: AACAACATGGAGCTGCAGAGG	R: GAAGTTGCCGTCTGCAAACAT
Caspase-3	F: TACCCTGAAATGGGCTTGTGT	R: GTTAACACGAGTGAGGATGTG

*RT-qPCR* reverse transcription quantitative polymerase chain reaction, *miR* microRNA, *GAPDH* glyceraldehyde-3-phosphate dehydrogenase, *Bcl*-*2* B cell leukemia 2, *Bax* Bcl-2 associated X, *R* reverse, *F* forward

The article "Bone mesenchymal stem cell-derived exosomal microRNA-29b-3p prevents hypoxic-ischemic injury in rat brain by activating the PTEN-mediated Akt signaling pathway" was retracted in 2020. Reasons: results that could not be reproduced; unreliable results or conclusions.

### Western blot analysis

Total proteins were extracted from tissues, cells, or exosomes by radioimmunoprecipitation assay lysis buffer (R0010, Beijing Solabio Life Sciences Co., Ltd., Beijing, China). The protein concentration was assessed through a bicinchoninic acid kit (20201ES76, Yeasen Biotechnology Co., Ltd., Shanghai, China). After being separated by polyacrylamide gel electrophoresis, the protein was transferred to a polyvinylidene fluoride membrane (Merck Millipore, Billerica, MA, USA) which was blocked in 5% BSA for one h at room temperature and then incubated with primary rabbit antibodies against TSG101 (ab30871, 1:1000), CD80 (ab109201, 1:1000), vascular endothelial growth factor A (VEGFA; ab46154, 1:1000), vascular endothelial growth factor receptor 2 (VEGFR2; ab11939, 1:1000), caspase 3 (ab13847, 1:1000), B cell leukemia 2 (Bcl-2; ab196495, 1:1000), Bcl-2 associated X (Bax; ab32503, 1:2000), Akt (ab8805, 1:1000) and p-Akt (ab38449, 1:1000), rat antibodies against CD63 (ab108950, 1:1000), and glyceraldehyde-3-phosphate dehydrogenase (GAPDH; ab8245, 1:5000). The membrane was then incubated with horseradish peroxidase-labeled goat anti-rabbit (ab205718, 1:10,000) or goat anti-mouse (ab6789, 1:5000) secondary antibody at room temperature for 1 h. The above antibodies were purchased from Abcam (Cambridge, UK). Bands were developed and band intensity was quantified using ImageJ 1.48u software (National Institutes of Health, Bethesda, MD, USA), with GAPDH used as an internal reference standard.

### Dual luciferase reporter gene assay

Reporter gene vectors of wild-type and binding site mutated (pGL3-PTEN-661 Wt/pGL3-PTEN-661 Mut and pGL3-PTEN-1703 Wt/pGL3-PTEN-1703 Mut) were constructed and transfected with miR-29b-3p mimic and pRL-TK (internal reference plasmid expressing luciferase of Renilla) in HEK293T cells (American Type Culture Collection, Manassas, VA, USA). Twenty-four hours later, cells were lysed according to the instructions of TransDetect Double-Luciferase Reporter Assay Kit (FR201-01, TransGen Biotech, Beijing, China) and the supernatant was collected to detect the activities of firefly (FL) and renilla (RL) luciferases in the Dual-Luciferase Reporter Assay System (E1910, Promega, Madison, Wis., USA). The ratio of FL/RL was used as the relative luciferase activity.

The article "Bone mesenchymal stem cell-derived exosomal microRNA-29b-3p prevents hypoxic-ischemic injury in rat brain by activating the PTEN-mediated Akt signaling pathway" was retracted in 2020. Reasons: results that could not be reproduced; unreliable results or conclusions.

### Tube formation assay

Cells were starved with serum-free medium for 24 h in cell suspension (1 × 10^5^ cells/mL) and cultured in 24-well plate coated with Matrigel (354234, Shanghai Shanran Biotechnology Co., Ltd., Shanghai, China) for 6 h. Capillary-like tube structures were identified under a Leica inverted phase contrast microscope (× 100). Tube length and branch point were calculated at five random fields using Image-Pro Plus 6.0 software.

### Immunohistochemistry

The expression of CD31 (ab24590, 1:100, Abcam, Cambridge, UK) and PTEN (ab170941, 1:100, Abcam, Cambridge, UK) was detected by routine immunohistochemical staining. The CD31 expression was observed under a microscope (IX53, Olympus Optical Co., Ltd., Tokyo, Japan) and microvessel density (MVD) was calculated by the method of Weidner [30]. CD31 was mainly expressed in the cytoplasm/membrane of endothelial cells, presenting as brown stain under the microscope. Five sections of each rat brain tissue were randomly selected for observation.

### Statistical analysis

SPSS 21.0 statistical software (IBM Corp. Armonk, NY, USA) was used for data analysis. All data were tested for normal distribution and homogeneity of variance using Levene’s test. The data conforming to the normal distribution were presented as mean ± standard deviation. Unpaired two-tailed *t* test was used for comparisons between two groups, and one-way analysis of variance (ANOVA) analysis was used for comparisons among multiple groups, followed by Tukey’s post-hoc tests. The difference was statistically significant when *p* < 0.05.

## Results

### Expression of miR-29b-3p is significantly decreased in the cerebral cortex of MCAO rats

A study has shown that miR-29b-3p is poorly expressed in intestinal ischemic injury models and reduces intestinal ischemic injury [15, 31]. However, the role of miR-29b-3p has remained uncertain in cerebral ischemic injury. We established the rat model with MCAO to investigate the molecular mechanism of miR-29b-3p in the ischemic brain injury. After 72 h, TTC staining showed that the brain of MCAO rats exhibited significant cerebral infarction compared with control sham rats (*p* < 0.05), suggesting that the ischemic brain injury model was successfully established (Fig. 1a, b). TUNEL staining was performed to detect the apoptosis in cerebral cortex. As shown in Fig. 1c, d, the apoptotic rate in the cortex of rats with MCAO was significantly increased (*p* < 0.05). Then we examined the apoptosis and angiogenesis-related proteins by Western blot analysis. As shown in Fig. 1e, f, the level of anti-apoptotic protein Bcl-2 was significantly inhibited in MCAO rats, while the pro-apoptotic protein Bax was significantly increased. Besides, the level of cleaved caspase-3 was also elevated, indicating that the apoptosis process was activated in the brain of MCAO rats. As for the angiogenesis-promoting proteins, we found that the levels of VEGFA and VEGFR2 were decreased significantly (Fig. 1e, f, *p* < 0.05). Immunohistochemistry staining revealed that the MVD indicated by CD31 staining was remarkably decreased in MCAO rats (Fig. 1g, h, *p* < 0.05). In addition, expression of miR-29b-3p was significantly downregulated in the infarcted brain tissue of MCAO rats versus that in the sham-operated rats (Fig. 1i, *p* < 0.05). These findings suggest that miR-29b-3p was decreased significantly in the brain of MCAO rats accompanied by increased cell apoptosis and decreased angiogenesis.

The article "Bone mesenchymal stem cell-derived exosomal microRNA-29b-3p prevents hypoxic-ischemic injury in rat brain by activating the PTEN-mediated Akt signaling pathway" was retracted in 2020. Reasons: results that could not be reproduced; unreliable results or conclusions.

**Fig. 1:** miR-29b-3p is downregulated in the cerebral cortex of MCAO rats. TTC staining (**a**) and the quantification (**b**) of the ischemic brain injury of MCAO rats. TUNEL staining (**c**) and the quantification (**d**) of the apoptosis in the cerebral cortex of MCAO rats (scale bar = 25 μm). **e**, **f** Western blot analysis of the expression of apoptosis- and angiogenesis-related proteins (Bcl-2, Bax, Cleaved caspase-3, VEGFA and VEGFR2) in the cerebral cortex. **g**, **h** CD31 immunofluorescence staining showed the microvessel density (MVD) in the cerebral cortex (scale bar = 25 μm). **i** RT-qPCR analysis of the expression of miR-29b-3p in the cerebral cortex of rats. *p < 0.05 vs. the sham group. The measurement data are expressed in the form of mean ± standard deviation. The comparison between the two groups was carried out by the independent sample *t* test. *n* = 7 rats in each group

### BMSCs reduce the neuron apoptosis and inhibit angiogenesis of BMECs exposed to OGD by releasing exosomes

Since exosomes derived from MSCs have been reported to protect against various kinds of disorders [32, 33], we sought to explore whether BMSC-derived exosomes (MSCs-Exos) have beneficial influences on OGD-induced injury to neurons and BMECs. OGD treatment was initially conducted in primary cultured cortical neurons and BMECs. Then these cells were co-cultured with BMSCs to measure relevant indexes. First, we observed that the apoptotic cell number was increased in OGD-stressed cortical neurons (Fig. 2a, b). Besides, the expression of Bax was enhanced, while the expression of Bcl-2 was decreased, whereas the activity of caspase-3 was activated in OGD cortical neurons (Fig. 2c, d). In addition, the levels of VEGFA and VEGFR2 were remarkably decreased (Fig. 2c, d), accompanied by inhibited tube formation of BMECs (Fig. 2e, f). Meanwhile, miR-29b-3p expression was significantly reduced in OGD cortical neurons (Fig. 2g). When co-cultured with BMSCs, the number of apoptotic cells was decreased in OGD cortical neurons, along with diminished expression of Bax and caspase-3 and promoted expression of Bcl-2. In addition, the tube formation of BMECs was significantly restored by the treatment, as evidenced by upregulated VEGFA and VEGFR2 expression. While the addition of GW4869 (an inhibitor of exosome secretion) led to no significant difference relative to cells treated with OGD (Fig. 2a–f). Finally, the expression of miR-29b-3p in OGD cortical neurons and BMECs co-cultured with BMSCs was significantly upregulated (Fig. 2g). On the other hand, GW4869 affected the delivery of exosomes, leading miR-29b-3p expression reduced to the same level as cells without co-culture. Therefore, BMSCs could reduce the neuron apoptosis and reverse the suppression in angiogenesis of BMECs induced by OGD by releasing exosomes.

The article "Bone mesenchymal stem cell-derived exosomal microRNA-29b-3p prevents hypoxic-ischemic injury in rat brain by activating the PTEN-mediated Akt signaling pathway" was retracted in 2020. Reasons: results that could not be reproduced; unreliable results or conclusions.

**Fig. 2:** BMSCs reduce the neuron apoptosis and inhibit angiogenesis of BMECs exposed to OGD by releasing exosomes. TUNEL staining (**a**) and the quantification (**b**) of apoptosis in cortical neurons (scale bar = 50 μm). **c**, **d** The protein expression and quantification of neuronal apoptosis- and angiogenesis-related proteins analyzed by western blot analysis. **e**, **f** Representative images and quantification of tube formation ability of BMECs (scale bar = 100 μm). **g** The expression of miR-29b-3p detected by RT-qPCR in cortical neurons and BMECs. *p < 0.05 vs. the control group. #*p* < 0.05 vs. the OGD + MSC group. The measurement data are expressed in the form of mean ± standard deviation. The comparison between the two groups was carried out by the independent sample *t* test. The experiment was repeated three times

### BMSCs transfer miR-29b-3p to neurons and BMECs through exosomes

Exosomes were extracted from culture medium of BMSCs at passage four, and the morphology was observed under a transmission electron microscopy (Fig. 3a). The size distribution of exosomes was confirmed by electron microscopy and dynamic light scattering (Fig. 3b), and the exosomes were positive for the MSC markers CD80, CD63, and TSG101, as verified by Western blot analysis (Fig. 3c). Thus, the exosomes were isolated successfully. Then, the BMSCs-derived exosomes were labeled with PKH-67 and added to the culture medium of cortical neurons or BMECs in the Transwell system. Four hours later, we observed a significant number of exosomes in neurons and BMECs (Fig. 3d). After 24 h, the expression of BMSC markers CD29, CD90, and CD105 was significantly increased in neurons and BMECs treated with BMSCs-derived exosomes. In addition, compared with untreated neurons and BMECs, the expression of miR-29b-3p was also significantly elevated in neurons and BMECs treated with BMSCs-derived exosomes (Fig. 3e, f). As shown in Fig. 3g, the reverse transcription quantitative polymerase chain reaction (RT-qPCR) results showed that miR-29b-3p expression was significantly upregulated in exosomes from BMSCs transfected with miR-29b-3p mimic and downregulated in exosomes from BMSCs transfected with miR-29b-3p inhibitor (*p* < 0.05). Similarly, after co-culture of BMSC-derived exosomes with neurons or BMECs, miR-29b-3p was significantly upregulated in neurons and BMECs co-cultured with exosomes from BMSCs overexpressing miR-29b-3p but downregulated after co-culture with exosomes from BMSCs transfected with miR-29b-3p inhibitor (Fig. 3h). Thus, the BMSCs could transfer exosome-shuttled miR-29b-3p into neurons or BMECs.

The article "Bone mesenchymal stem cell-derived exosomal microRNA-29b-3p prevents hypoxic-ischemic injury in rat brain by activating the PTEN-mediated Akt signaling pathway" was retracted in 2020. Reasons: results that could not be reproduced; unreliable results or conclusions.

**Fig. 3:** The exosomes derived from BMSCs carry miR-29b-3p. **a** Morphologic observation of the exosomes under a transmission electron microscopy (scale bar = 200 nm). **b** Particle size distribution measured by DLS. **c** The protein expression of TSG101, CD80 and CD63 in exosomes from BMSCs detected by western blot analysis. **d** The PHK-67-labeled exosomes in neurons and BMECs observed under a fluorescence microscope (scale bar = 50 μm). **e**, **f** The expression of BMSCs marker proteins and miR-29b-3p in neurons and BMECs treated with BMSCs-secreted exosomes detected by RT-qPCR. **g**, **h** The expression of miR-29b-3p in neurons and BMECs treated with BMSCs-secreted exosomes containing miR-29b-3p mimic or inhibitor, as detected by RT-qPCR. *p < 0.05 vs. the control group or the OGD group, #*p* < 0.05 vs. the OGD + BMSCs group. The measurement data are expressed in the form of mean ± standard deviation. The comparison between the two groups was carried out by the independent sample *t* test. Comparison among multiple groups was conducted using one-way analysis of variance, followed by Tukey’s post hoc test. The experiment was repeated three times

### BMSCs-derived exosomal miR-29b-3p attenuates neuronal apoptosis and promotes BMEC angiogenesis

To identify whether BMSCs-derived exosomal miR-29b-3p is related to regulation of neuronal apoptosis and BMEC angiogenesis, neurons and BMECs were treated with BMSCs-derived exosomes expressing NC mimic, miR-29b-3p mimic, NC inhibitor, or miR-29b-3p inhibitor, and then collected for further analysis. The TUNEL staining showed that the apoptosis of the neurons treated with MSCs-Exo miR-29b-3p mimic was lower than that of neurons treated with MSCs-Exo NC mimic, and that apoptosis was significantly increased in neurons treated with MSCs-Exo miR-29b-3p inhibitor compared with those treated with MSCs-Exo NC inhibitor (Fig. 4a, b). Furthermore, Western blot analysis confirmed that the expression of Bcl-2, VEGFA, and VEGFR2 in the cortical neurons was upregulated by MSCs-Exo miR-29b-3p mimic, and that the expression of Bax and cleaved caspase-3 was inhibited. By contrast, co-culture with MSCs-Exosomes containing miR-29b-3p inhibitor contributed to diminished Bcl-2, VEGFA and VEGFR2, while promoting Bax and cleaved caspase-3 expression in cortical neurons (Fig. 4c, d). Tube formation assay revealed that the number of branch points was significantly increased following treatment of MSCs-Exo miR-29b-3p mimic, while the number of branch points after MSCs-Exo miR-29b-3p inhibitor was significantly reduced (Fig. 4e). Therefore, the exosomes released from BMSCs overexpression miR-29b-3p was able to ameliorate the neuron apoptosis and reverse suppression in BMEC angiogenesis caused by OGD treatment.

The article "Bone mesenchymal stem cell-derived exosomal microRNA-29b-3p prevents hypoxic-ischemic injury in rat brain by activating the PTEN-mediated Akt signaling pathway" was retracted in 2020. Reasons: results that could not be reproduced; unreliable results or conclusions.

**Fig. 4:** miR-29b-3p in BMSC-derived exosomes ameliorates OGD-induced cell injury. **a**, **b** Apoptosis of cortical neurons after treated with BMSC-derived exosomes detected by TUNEL staining (scale bar = 50 μm). **c**, **d** The expression of neuronal apoptosis- and BMECs angiogenesis-related proteins analyzed by western blot analysis. **e** Representative images and quantification of tube formation ability of BMECs after treated with BMSC-derived exosomes (scale bar = 100 μm). *p < 0.05 vs. the NC mimic group, #*p* < 0.05 vs. the NC inhibitor group. The measurement data are expressed as mean ± standard deviation. The comparison between the two groups was carried out by the independent sample *t* test. The experiment was repeated in triplicate

### miR-29b-3p targets PTEN to decrease neuron injury induced by OGD

The potential binding sites between miR-29b-3p and PTEN gene were predicted using TargetScan (http://www.targetscan.org), showing that miR-29b-3p could bind to the sequences 661-688 and 1703-1709 of PTEN gene (Fig. 5a). Dual luciferase reporter gene assay (Fig. 5b) showed that the relative luciferase activity of PTEN 661-WT was decreased (*p* < 0.05), while there was no significant difference in luciferase activity of PTEN 1703-WT and PTEN-MUT co-transfected with miR-29b-3p mimic (*p* > 0.05), suggesting that miR-29b-3p could specifically bind to the 661 site of PTEN gene. The level of PTEN in response to miR-29b-3p overexpression in cortical neurons and BMECs (Fig. 5c, d) showed that, upon miR-29b-3p overexpression, PTEN was significantly downregulated at both mRNA and protein levels in neurons and BMECs (*p* < 0.05). These data consistently showed that PTEN could be a target gene of miR-29b-3p.

The article "Bone mesenchymal stem cell-derived exosomal microRNA-29b-3p prevents hypoxic-ischemic injury in rat brain by activating the PTEN-mediated Akt signaling pathway" was retracted in 2020. Reasons: results that could not be reproduced; unreliable results or conclusions.

**Fig. 5:** PTEN is targeted and negatively regulated by miR-29b-3p, and the silencing of PTEN attenuates the OGD-induced injury on neurons and BMECs. **a** The binding sites between miR-29b-3p and PTEN gene predicted by TargetScan website. **b** The regulation of miR-29b-3p on PTEN gene transcription verified by dual luciferase reporter gene assay. **c** mRNA level of PTEN was detected by RT-qPCR in neurons and BMECs infected with lentivirus harboring miR-29b-3p. **d** The protein expression of PTEN detected by western blot analysis in neurons and BMECs infected with lentivirus harboring miR-29b-3p. The mRNA **e** and protein **f** expression of PTEN were elevated in MCAO rats and OGD cells. **g**, **h** Western blot analysis of neuronal apoptosis- and BMECs angiogenesis-related proteins in neurons and BMECs infected with lentivirus harboring miR-29b-3p and or PTEN shRNA. **i** The tube formation ability of BMECs infected with lentivirus harboring miR-29b-3p and or PTEN shRNA (scale bar = 100 μm). *p < 0.05 vs. the PGL-3 vector group, NC group, sham group, control group or Lv-vector group. #*p* < 0.05 vs. the Lv-miR-29b-3p group or Lv-sh-PTEN group. *Lv* Lentivirus. The measurement data are expressed as mean ± standard deviation. The comparison between the two groups was carried out by the independent sample *t* test. Comparison among multiple groups was conducted using one-way analysis of variance, followed by Tukey’s post hoc test. The experiment was repeated three times

Further, we probed into the effect of PTEN on ischemic brain injury. First, we found that the expression of PTEN was significantly upregulated in MCAO rats and OGD cells at both mRNA and protein levels with RT-qPCR and Western blot analysis (Fig. 5e, f). OGD neurons or BMECs were infected with lentivirus harboring miR-29b-3p and/or PTEN shRNA. As shown in Fig. 5g, h, the expression of Bax and cleaved caspase-3 was significantly decreased and Bcl-2 was upregulated in neurons after PTEN was downregulated, while the expression of angiogenesis-promoting proteins (VEGFA and VEGFR2) was significantly increased in BMECs, findings in line with the effects of miR-29b-3p overexpression. In addition, the silencing of PTEN could also enhance tube formation induced by miR-29b-3p overexpression in BMECs, and further inhibit pro-apoptosis gene expression (Fig. 5i). All of these results suggested that miR-29b-3p overexpression promoted tube formation of BMECs and repressed neuronal apoptosis by targeting PTEN.

The article "Bone mesenchymal stem cell-derived exosomal microRNA-29b-3p prevents hypoxic-ischemic injury in rat brain by activating the PTEN-mediated Akt signaling pathway" was retracted in 2020. Reasons: results that could not be reproduced; unreliable results or conclusions.

### BMSC-derived exosomal miR-29b-3p activates the Akt signaling pathway via targeting PTEN

As PTEN was reported to negatively regulate Akt signaling pathways [34], we tested whether Akt participated in the regulation of miR-29b-3p in a co-culture system of OGD cortical neurons and BMECs with BMSCs. The phosphorylation of Akt was elevated in OGD cortical neurons and BMECs when co-cultured with miR-29b-3p expressed BMSCs (Fig. 6a, b, e, f). Whereas, the phosphorylation of Akt was suppressed by miR-29b-3p inhibitor, further supporting that miR-29b-3p blocked the activation of the Akt signaling pathway. Upon silencing of PTEN, the phosphorylation of Akt was enhanced in both OGD cortical neurons and BMECs (Fig. 6c, d, g, h). Collectively, miR-29b-3p inhibits PTEN expression and further promotes Akt activation.

**Fig. 6:** miR-29b-3p activates the Akt signaling pathway. Akt phosphorylation was detected in neurons infected with lentivirus harboring miR-29b-3p mimic or miR-29b-3p inhibitor (**a**, **b**), or PTEN shRNA (**c**, **d**). Akt phosphorylation was detected in BMECs infected with lentivirus harboring miR-29b-3p mimic or miR-29b-3p inhibitor (**e**, **f**), or PTEN shRNA (**g**, **h**). *p < 0.05 vs. the NC mimic group or vector group. The measurement data are expressed as mean ± standard deviation. The comparison between the two groups was carried out by the independent sample *t* test. The experiment was repeated three times

### BMSC-derived exosomal miR-29b-3p alleviates the brain injury in MCAO rats

Finally, we examined whether BMSC-derived exosomes play a beneficial role in the brain injury of MCAO rats. One hour after surgery, exosomes from untreated BMSCs (MSCs-Exo) or BMSCs expressing miR-29b-3p agomir (MSCs-Exo-miR-29b-3p agomir) were injected stereotactically into the brain. As shown in Fig. 7a, b, 2 weeks later, the volume of brain injury in the MSCs-Exo and MSCs-Exo-miR-29b-3p agomir groups was significantly less than that in the saline group, and the injury in the MSCs-Exo-miR-29b-3p agomir group was significantly less than that in the MSCs-Exo group. Besides, compared with the saline group, miR-29b-3p was significantly upregulated in the MSCs-Exo and MSCs-Exo-miR-29b-3p agomir groups, while the PTEN was significantly downregulated as detected by both RT-qPCR and immunohistochemistry staining. Specifically, the alteration of miR-29b-3p and PTEN was more highly significant in the MSCs-Exo-miR-29b-3p agomir group (Fig. 7c–e). The apoptosis- and angiogenesis-related proteins (Fig. 7f, g) and TUNEL staining showed that the apoptotic level of the injured sites was attenuated in the MSCs-Exo and MSCs-Exo-miR-29b-3p agomir groups, which was more prominent in the MSCs-Exo-miR-29b-3p agomir group. In addition, the expression of Bcl-2, VEGFA ,and VEGFR2 was enhanced, while that of Bax and cleaved caspase-3 was reduced in the MSCs-Exo and MSCs-Exo-miR-29b-3p agomir groups; the difference was more pronounced in BMSC-exosome-miR-29b-3p agomir group (Fig. 7h, i). In accordance, the immunohistochemistry staining of CD31 showed that angiogenesis was increased in the MSCs-Exo and MSCs-Exo-miR-29b-3p agomir groups, and the angiogenesis promotion was significantly more notably in the MSCs-Exo-miR-29b-3p agomir group (Fig. 7j, k). The results showed that BMSC-derived exosomes could alleviate the brain injury in MCAO rats, and that miR-29b-3p agomir could further promote the beneficial effects of BMSC-derived exosomes in the brain injury.

The article "Bone mesenchymal stem cell-derived exosomal microRNA-29b-3p prevents hypoxic-ischemic injury in rat brain by activating the PTEN-mediated Akt signaling pathway" was retracted in 2020. Reasons: results that could not be reproduced; unreliable results or conclusions.

**Fig. 7:** Exosomal miR-29b-3p from BMSCs ameliorates brain injury in MCAO rats. The brain of MCAO rats was injected with exosomes from untreated BMSCs or miR-29b-3p agomir over-expressed BMSCs. **a**, **b** The volume of brain injury shown by TTC staining. **c** The mRNA expression of PTEN and miR-29b-3p expression determined by RT-qPCR. **d**, **e** The protein expression of PTEN shown by immunohistochemistry staining (scale bar = 50 μm). **f**, **g** The apoptosis shown by TUNEL staining (scale bar = 50 μm). **h**, **i** The protein expression of apoptosis and angiogenesis-related genes measured by western blot analysis. **j**, **k** The immunohistochemical staining of CD31 and MVD in brain tissues (scale bar = 25 μm). *p < 0.05, vs. the saline group. #*p* < 0.05, vs. the MSCs-Exo group. The measurement data are expressed as mean ± standard deviation. The comparison among multiple groups was conducted using one-way analysis of variance, followed by Turkey’s post hoc test. The experiment was repeated three times, with *n* = 7 in each group

## Discussion

MSCs have gained much interest in the therapy for various disorders and have also shown augmented protection in the treatment of neonatal hypoxic-ischemic brain injury [35]. Recently, exosomes derived from MSCs have been found to carry various kinds of mediators, miRNAs and proteins, which can mediate the function of MSCs [10, 36, 37]. Besides, the reports of altered expression of miRNAs in hypoxic-ischemic brain injury suggest that miRNAs may participate in the pathogenesis of this model [38]. Based on this fact, we explored the role of miR-29b-3p in the BMSC-derived exosomes and in neuronal apoptosis and BMEC angiogenesis in the hypoxic-ischemic brain injury. Collectively, the data of the study revealed that BMSC-derived exosomal miR-29b-3p could indeed suppress neuronal apoptosis and promote angiogenesis of BMECs through the downregulation of PTEN and activation of Akt signaling pathway.

The article "Bone mesenchymal stem cell-derived exosomal microRNA-29b-3p prevents hypoxic-ischemic injury in rat brain by activating the PTEN-mediated Akt signaling pathway" was retracted in 2020. Reasons: results that could not be reproduced; unreliable results or conclusions.

First, we found that miR-29b-3p was significantly downregulated and PTEN was upregulated in MCAO rats, and OGD neurons and BMECs. The miR-29 family consists of miR-29a, miR-29b (b1 and b2 which are identical mature miRNAs), and miR-29c, with the mature miRNAs differing only in two or three bases. The expression of miR-29b-3p was found to be increased in osteoarthritis compared to the healthy neck-of-femur [39]. Indeed, miR-29b-3p potentiates chondrocyte apoptosis and facilitates the occurrence and progression of osteoarthritis [40]. Also, BMSC-specific overexpression of miR-29b-3p induced insulin resistance in young mice [41]. A previous study showed that miR-29b-3p protects against hypoxia-induced cell apoptosis [42]. PTEN is generally understood to be tumor-inhibiting protein but also plays important roles in neurological diseases [43]. For example, knockdown of PTEN was reportedly able to protect mouse brain from ischemic injury [44]. Second, we found that the apoptosis was increased in MCAO rats and OGD cells, and in BMSC-derived exosomes, whereas exosomal delivery of miR-29b-3p could inhibit the apoptosis in these models. The overexpression of miR-29b-3p in OGD neurons or BMECs decreased the expression of Bax and cleaved caspase 3 and upregulated Bcl-2, confirming the inhibition of miR-29b-3p on cell apoptosis.

Emerging data support a helpful role for angiogenesis and neurovascular repair, together with a close interaction between angiogenesis and neurogenesis [45]. Ischemic stroke manifests as an ischemic core where neuron death proceeds rapidly, which is surrounded by a vulnerable peri-infarct area, whereas angiogenic blood vessels near the infarct function as a scaffold for neuronal progenitors, empowering neurons to migrate toward the peri-ischemic regions [46]. Neurogenesis and angiogenesis could thus be viewed as a complex and dynamic coupling with complex cross-talk between neurons and endothelial cells through vascular endothelial growth factor (VEGF), neurotrophins, as well as their cognate receptors on both neurons and endothelial cells [47]. Specifically, the 15-LO-1/15-HETE system presents a potential approach for aiding neurobehavioral recovery after cerebral ischemic stroke, a beneficial effect mediated by upregulation of VEGF and subsequent promotion of angiogenesis in the ischemic brains [48]. Exosomal signaling during hypoxia regulates angiogenesis and migration of MECs [49], and recent research shows that hypoxia stimulates the release of exosomes in various tumor types, culminating in the activation of vascular cells and angiogenesis [50]. According to a recent review, cell-based and cell free (exosomes, extracellular vesicles, microRNAs) therapies have already been applied successfully for angiogenesis-mediated tissue regeneration and have great potential for treating ischemic heart disease, brain stroke, as well as bone defects [51]. Furthermore, exosome-derived communication between endothelial cells and cardiomyocytes shows the potential for induction of local neo-vascularization during cardiac injury, and furthermore, cardiomyocyte-derived exosomes carry a broad repertoire of miRNAs and proteins under conditions of glucose deprivation [52]. In another example, exosomes derived from miR-126-modified MSCs facilitated the angiogenesis and migration of human umbilical venous endothelial cells after spinal cord injury [53]. Besides, upregulation of miR-29b plays a promotive role in ischemia-induced angiogenesis [54], indicating that miR-29b-3p is a promising factor in the treatment of hypoxic-ischemic brain injury. In this study, we revealed that declining cerebral levels of miR-29b-3p in MCAO rat brain was related to decreased angiogenesis, as indicated by the deregulation of VEGFA, VEGFR2 and CD31. In addition, the injection of BMSCs-derived exosomes containing miR-29b-3p mimic could ameliorate the suppression of angiogenesis in MCAO rats, further supporting miR-29b-3p to be a potential factor for the treatment of hypoxia-ischemia brain injury.

The article "Bone mesenchymal stem cell-derived exosomal microRNA-29b-3p prevents hypoxic-ischemic injury in rat brain by activating the PTEN-mediated Akt signaling pathway" was retracted in 2020. Reasons: results that could not be reproduced; unreliable results or conclusions.

Finally, we found that negative regulation of PTEN and activation of Akt mediated the effects of miR-29b-3p on the amelioration of brain injury caused by hypoxic-ischemia in the present models. The suppression of PTEN could activate the Akt signaling pathway and also mediated protection against ischemic neuronal death [43]. Besides, the inhibition of PTEN and activation of Akt by baicalen can suppress oxidant stress and scavenge free radicals in the ischemia/reperfusion injury model [44]. Finally, we note that the PI3K/Akt signaling pathway can accelerate angiogenesis after ischemic stroke [55]. Our present report further confirmed the critical role of PTEN and Akt pathway in the pathogenesis and recovery of hypoxic-ischemic brain injury.

## Conclusion

These findings provided new insights into the pathogenesis of hypoxic-ischemic brain injury, showing that miR-29b-3p was downregulated in MCAO rats and neurons under exposure to OGD. Besides, miR-29b-3p delivered in exosomes from BMSCs accelerated angiogenesis of BMECs and hindered neuronal apoptosis after ischemic stroke via targeting PTEN and activating the Akt signaling pathway (Fig. 8). Thus, present results show that miR-29b-3p may well present a potential therapeutic target in the experimental treatment of hypoxic-ischemic brain injury.

The article "Bone mesenchymal stem cell-derived exosomal microRNA-29b-3p prevents hypoxic-ischemic injury in rat brain by activating the PTEN-mediated Akt signaling pathway" was retracted in 2020. Reasons: results that could not be reproduced; unreliable results or conclusions.

**Fig. 8:** BMSC-derived exosomal miR-29b-3p suppresses neuronal apoptosis and promotes BMECs angiogenesis through the downregulation of PTEN and activation of the Akt signaling pathway

### Affiliated results

#### Immunofluorescence assay

After stable growth, cells were fixed with 4% paraformaldehyde at ambient temperature for 30 min. After permeabilization and sealing, cells were incubated with primary mouse antibodies against CD90 (ab225, 1:1000), CD105 (ab11414, 1:1000), Vimentin (ab8978, 1:1000), E-cadherin (ab1416, 1:1000), CD31 (ab24590, 1:1000), and rabbit antibodies against CD44 (ab157107, 1:1000), NeuN (ab177487, 1:300), and MAP2 (ab32454, 1:1000) overnight at 4 °C. Subsequently, the cells were incubated with fluorescent secondary antibody goat anti-mouse (ab6785, 1:1000) (green) or goat anti-rabbit (ab150075, 1: 000) (red) at ambient temperature for 60 min in the dark. All of the above antibodies were purchased from Abcam (Cambridge, UK). The cells were stained with DAPI for 10 min at ambient temperature and sealed with a sealing agent (36,308 ES11, Yeasen Biotechnology Co., Ltd., Shanghai, China), and finally observed under a fluorescence microscope (BX53, Olympus, Tokyo, Japan).

#### Primary BMSCs, cortical neurons, and BMECs were successfully isolated

BMSCs at passage 4 presented fibroblasts-like appearance as shown in Additional file 1: Figure S1A. Immunofluorescence assay displayed that BMSCs were positive for CD90, CD44, CD105, and negative for E-cadherin and Vimentin (Additional file 1: Figure S1B), suggesting successful isolation of BMSCs.

The cultured cortical neurons adhering to the wall 3 h after seeding were mostly round and sphere-shaped, with a few protrusions. On the sixth day, the neurons formed a complex neuroid (Additional file 1: Figure S1C). The expression of neuron marker nuclear proteins NeuN and MAP2 was detected by cellular immunofluorescence. The results showed that neurons were positive for NeuN (Additional file 1: Figure S1D), suggesting successful isolation of cortical neurons.

BMECs at the third day presented a typical flagstone-like structure and a “vortex-like distribution” (Additional file 1: Figure S1E). The CD31 immunofluorescence assay confirmed the successful isolation of BMECs (Additional file 1: Figure S1F).

## Supplementary information

**Additional file 1.Figure S1.** Isolation and identification of primary BMSCs, cortical neurons and BMECs. Light microscopic observation (A; scale bar = 50 μm) and immunofluorescence staining (B; scale bar = 25 μm) of CD90, CD44, CD105, E-cadherin and Vimentin in primary BMSCs. Light microscopic observation (C; scale bar = 50 μm) and immunofluorescence staining (D; scale bar = 50 μm) of NeuN and MAP2 in primary cortical neurons. Microscopic observation (E; scale bar = 50 μm) and CD31 immunofluorescence staining (F; scale bar = 25 μm) of BMECs. (EPS 27896 kb)

The article "Bone mesenchymal stem cell-derived exosomal microRNA-29b-3p prevents hypoxic-ischemic injury in rat brain by activating the PTEN-mediated Akt signaling pathway" was retracted in 2020. Reasons: results that could not be reproduced; unreliable results or conclusions.

## Data Availability

The datasets generated/analyzed during the current study are available.
